# Influence of Multiple Music Styles and Composition Styles on College Students' Mental Health

This article has been retracted.

**DOI:** 10.1155/2022/6167197

**Published:** 2022-07-12

**Authors:** Ququ Zheng, Vincent Lam

**Affiliations:** ^1^School of Music, Shanghai University, Shanghai City 200444, China; ^2^Amazon Music, 525 Market St FL19, San Francisco, CA 94105, USA

## Abstract

The purpose is to reduce students' psychological pressure and improve their quality of study and life. Here, 400 language-impaired students in the public elective psychology course at Northwestern University and the undergraduate psychology class at Xi'an Foreign Studies University in the 2018-2019 academic year are randomly selected as the research objects for this music psychology experiment. The students were divided into different experimental groups using the Questionnaire Survey (QS) method to analyze the students' psychological reactions to Baroque, classical, and romantic music styles. Then, it further discusses the students' emotional response and audiovisual synaesthesia, as well as their recognition and choice of music style. The results show that there are significant differences in the same emotional response intensity of the subjects to different styles of music creation. The music expression is consistent with the actual feelings of the subjects. The tonality and color density of audiovisual synaesthesia vary with the style of music creation. Different music creation styles generate different associations in students' minds, thus showing different psychological reactions. The QS results indicate that soft and soothing music can relieve students' learning pressure most, while music with a strong sense of rhythm and vitality has no significant effect. Therefore, different music creation styles affect students' learning pressure differently. This work discusses the influence of different music creation styles on the mental health of contemporary college students and provides a reference for music therapy to relieve students' learning pressure in the future.

## 1. Introduction

The 21^st^ century marks rapid information globalization, with which the pace of social progress is speeding up, the social competition is getting fierce, and the mental stress of the language-impaired students is increasing overwhelmingly. Against such a social background, the mental quality of language-impaired students concerns not only their personal problems but also the overall quality of the whole society, as well as the future talent training and social development. Music psychology originated in Germany in the 19th century. The research object and content of music psychology is the relationship between music and people's psychological activities [1]. It is a new frontier cross-disciplinary in musicology and psychology. Following over a century of development, music psychology has evolved into a discipline beneficial to human physical and mental health [2], with wide real-life applications [3]. Positive psychology has caught the eyes of the public from the early 21^st^ century and has developed into a new psychological school. After all, positive psychology is closely related to human well-being ([4]); [5]). There have been studies on the relationship between musicology and psychology in music therapy and music psychology, as well as the effect of music on human physiology and psychological emotion, proving that the relationship between music and emotions plays a significant positive role in the treatment of college students' mental health [6]. Apart from a comfortable learning and scientific research environment for language-impaired students to develop self-dependent knowledge-learning abilities and skills, special education schools should also create a pleasant living and ideological environment for them to cultivate their humanistic tastes and ideological and moral standards, thereby helping them establish correct life values, world outlook, healthy personalities [7, 8]. Only through comprehensive psychophysiological cultivation can these special groups of students develop healthily, based on which the overall national quality can be promoted and social progress can be further advanced [9]. Meanwhile, the study of psychotherapy combined with different types of global music reveals that different music styles play a positive role in the physical and mental health, interpersonal relationships, social communication process, and life interests of language-impaired students, which is of great reference value for the music therapy research on language-impaired students. Therefore, targeted psychotherapy can be conducted for language-impaired students by combining all kinds of music data around the world. Bettis et al. [10] studied music therapy and psychology and pointed out that the relationship between music and psychology played a positive role in the physiology, mental health, interpersonal relationship, social interaction process, and emotions of language-impaired students [10]. Lattie et al. [11] argued that the relationship between music and psychology could enhance the treatment of the mental health of language-impaired students. Therefore, music therapy could effectively solve the mental health problems of language-impaired students [11]. Language impairment includes specific speech dysarthria (a specific speech developmental disorder, children with which show lower language useability than that of their intellectual age but with normal language skills); expressive language disorder (a specific speech and language developmental disorder, children with which show a significantly lower oral application ability with expressive language than that of their intellectual age but with a normal language comprehension ability and accompanied by pronunciation abnormality sometimes); and perceptual language disorder (a specific language development disorder, children with which show a lower language understanding than that of their intellectual age and almost all suffer from a significant language impairment, usually accompanied by an abnormal speech development).

Music therapy has shown significant prospects in mental health treatment. For example, music therapy has played a positive role in adjusting students' emotions [12], cultivating students' healthy emotions, eliminating interpersonal barriers, and improving the development of students' innovative thinking and innovation ability [13, 14] through mental health education and psychological counseling courses, as well as the prevention and treatment of students' mental health problems. These measures, in turn, can help form systematic theoretical support for music therapy, to better guide mental health education for language-impaired students, and further promote the development of music therapy in college mental health education [15]. At present, there is little research on which type of music can maximize the effect of music psychotherapy. With the continuous development of digital multimedia technology, music resources are substantially enriched; thus, from the user's point of view, an effective mechanism to obtain their preferable songs, or, from the physician's point of view, a feasible approach to pick out songs for music psychotherapy from the voluminous music library have both become difficult problems. Given this dilemma, the personalized music recommendation system came into being, which, however, has presented uneven recommendation effects and some defects despite many practical applications. Recent years have also witnessed the emergence of an efficient Deep Learning (DL) method: Convolutional Neural Network (CNN) [16], which has attracted extensive attention and, thus, seen wide applications in many fields, such as image recognition and Natural Language Processing (NLP), thereby achieving better results than traditional Machine Learning (ML) algorithms [17]. The CNN model is different from the traditional Artificial Neural Network (ANN) model, with the classification and prediction completely sealed within a black box; its weights trained by a Back-Propagation (BP) algorithm and its network parameters are obtained through continuous optimization; thus, the CNN model can be regarded as a feature extractor for automatic synthesis. Thereupon, this paper presents a CNN-based music recommendation system.

The above literature review summarizes the existing problems in music recommendation systems [18]. Specifically, the existing music psychology does not include music enhancement of positive psychological emotions, music alleviation of negative psychological emotions, and music identification research [19, 20]. The above experts and scholars mainly analyzed the impact of different music styles on students' mental health from the perspectives of music psychology, positive psychology, language barriers, and special education. They have enriched the theoretical basis in this field. The deficiency lies in that they have not clarified how to alleviate and treat the mental health problems of college students in the future, and it lacks certain feasibility. Additionally, under increasing diverse music types, there are few studies on how to select appropriate music types to achieve the best effect of psychological adjuvant therapy. Therefore, based on the previous studies, the relevant research results of music psychology and positive psychology are cited. Following literature research and empirical investigation, the enhancement effect of positive psychology and the alleviation effect of negative psychology is explored in language-impaired students' mental health through music therapy. At the same time, by collecting the historical behavior information of music users, this paper constructs the user music dataset for model training and testing and proposes a CNN-based music recommendation system. Innovatively, music is applied to the mental health treatment of contemporary language-impaired students, which is believed to provide a breakthrough for the mental health development of language-impaired students; moreover, a CNN-based music recommendation system for psychotherapy is established, and the network model structure used in the system experiment is designed based on the typical CNN model. Finally, the model training and optimization parameters are compared and selected. This work has some innovative points. Based on the previous research on music psychology, it takes the relevant research results of music psychology and positive psychology as the theoretical basis and researches music therapy to enhance the positive psychology of language-impaired students and alleviate their negative psychology through literature research and empirical investigation. The finding provides a research theory with reference significance for cultivating and educating the mental health of language-impaired students.

## 2. Research Methods of the Influence of Music Style on the Mental Health of Language-Impaired Students

### 2.1. Research Topics and Methods

#### 2.1.1. Subjects

About 400 language-impaired students are randomly selected from the public elective course of the psychology at Northwest University from 2018 to 2019 academic year and the undergraduate psychology course of Xi'an Foreign Languages University for music psychological experiments.

#### 2.1.2. Related Literature Method

It summarizes and discusses the previous achievements of music psychology and related literature review. Here, the domestic and international research results are reviewed for music psychology, music therapy, and the mental health of language-impaired students. Then, based on previous research results, the shortcomings of previous studies are innovatively explored [21].

#### 2.1.3. Case Interview Method

Here, case interview research is randomly conducted on language-impaired students to sort out students' psychological manifestation of stimulus music sources, including music cognition, imagination, will, emotion, and music personality, thereby analyzing the individual self-feelings and collective feelings of each kind of music [22].

#### 2.1.4. Theoretical Analysis

A global music database is established based on information globalization technology, and the positive effects of different music styles are analyzed on students' psychotherapy. Then, theoretical analysis, induction, and deduction are carried out through the music psychosomatic regulation experiment, and working principles of music psychotherapy and the positive role of music are theoretically explained from the perspective of personality psychology and positive psychology [23].

### 2.2. QS (Questionnaire Survey) Method

Here, several experimental scales, including the music positive psychological enhancement scale, music psychosomatic adjustment scale, and music negative psychological alleviation scale, are designed, through which the randomly selected subjects are surveyed. Then, the Likert five-point scale is used for scoring standards, specifically, 1 = lowest, 2 = lower, 3 = medium, 4 = higher, and 5 = highest [24, 25]. The first part is the empirical study of music enhancement on the subjects' 10 positive emotions (joy, quiet, gratitude, hope, interest, harmony, pride, incentive, optimism, and kindness), for which 16 music works are selected. Afterward, the music enhancement of each positive emotion and the comprehensive enhancement of positive emotions are evaluated and empirically analyzed under the stimulation of different music works [26]. Thus, the structural equation model of music psychology is constructed to improve positive psychological quality [27]. The second part is the empirical study on the music alleviation of 10 negative emotions (sadness, anger, worry, complaint, pain, anxiety, abomination, fear, loneliness, and sorrow). Similarly, 16 music works are selected [28]. Subsequently, the music alleviation of each negative emotion and the comprehensive alleviation of negative emotions are evaluated and empirically analyzed under the stimulation of different music works [29, 30]. Thus, a structural equation model of music psychology is constructed to alleviate negative emotions. The third part is the empirical study on the interaction effect of music's psychological effect on negative emotions and positive emotions. The objective is to establish the structural equation model of nine kinds of music's psychological interaction effects through empirical analysis to enhance positive emotion and alleviate negative emotion [31]. Among them, there are 16 kinds of music repertoire, including positive emotion enhancement, negative emotion alleviation, and the correlation effect between positive emotion enhancement and negative emotion alleviation [32].

### 2.3. Statistical Methods and Modeling

Here, the American social science statistical software package SPSS25.0 is adopted for data processing on the survey subjects. Specifically, the statistical methods include variable correlation analysis, basic data description analysis, and multiple regression analysis. The reliability of the QS is tested using Cronbach's *α* coefficient. The Cronbach's *α* coefficient of the QS is 0.835, and the reliability of the QS is high. KMO (Kaiser Meyer Olkin) and Bartlett spherical test can test the validity of the QS. The KMO value of the QS is between 0.9 and 1, and the Bartlett spherical test is significant (*P* < 0.05), so the validity is high [31]. The calculation of Cronbach's *α* coefficient is expressed as in

(1) $$\begin{array}{c} \alpha =\frac{nr}{\left[\left(n-1\right)r+1\right]}. \end{array}$$

Regression analysis is based on massive amounts of observation data; the regression relationship function (regression equation) is established through the mathematical statistics method for dependent variables and independent variables. Regression analysis is a predictive modeling technology that studies the relationship between the dependent variable (target) and the independent variable (predictor), as well as the relationship between the dependent variable and the uncertainty of the independent variable, namely, correlation. Thus, regression analysis is usually used for prediction analysis, time series modeling and the excavation of causal relationships between variables. Linear Regression is a well-known modeling technique that is preferred in learning prediction models. In Linear Regression, the dependent variable is continuous, the independent variable can be continuous or discrete, and the nature of the regression line is linear. Linear Regression establishes a relationship between the dependent variable (*Y*) and one or more independent variables (*X*) with the best fitting line (regression line), as expressed in

(2) $$\begin{array}{c} Y=a+b\times X+e. \end{array}$$

In Equation (2), *a* represents the intercept, *b* indicates the slope of the straight line, and *e* denotes the error term. Equation (2) can predict the value of the target variable according to the given prediction variables.

Subsequently, the American structural equation modeling software AMOS7.0 is chosen to fit the structural equation prediction model of music performance-positive and negative emotional experience for language-impaired students (Li et al., 2017). The structural equation prediction model is shown in Figure 1.

In Figure 1, ten music works are selected for an empirical study on the music's enhancement effect on ten positive emotions and the alleviation effect on ten negative emotions. The ten positive emotions are joy, quiet, gratitude, hope, interest, harmony, pride, incentive, optimism, and kindness. The ten negative emotions are sadness, sorrow, anger, complaint, anxiety, pain, fear, worry, loneliness, and abomination. These emotions are evaluated and analyzed to build a “structural equation model of music psychology enhancing positive psychological quality.”

### 2.4. CNN

So far, CNN has seen wide applications in image, text, and other recommendation systems, among which the CNN-based music recommendation system is the focus of this paper; in essence, the CNN-based music recommendation system is a hybrid model based on music content and user historical behaviors. The core idea of the recommendation algorithm is to use CNN to predict the implicit features of music, obtain the low-dimensional vector representation of music features, and then combine the implicit representation of user preferences to generate reasonable Top N recommendations for relevant users. The music features extracted from the audio signal can essentially express the characteristics of music, better fit human's intuitive feeling of the music, and effectively avoid the cold start problem. This section will describe the related contents in implementing recommendation algorithms, such as latent factor model, matrix decomposition, audio feature representation, and CNN model architecture design to achieve a better recommendation effect.

CNN is a kind of deep-structured feedforward neural network (NN) with convolution operation. The research on CNN can be traced back to the 1980s and 1990s. TDNN and LeNet-5 are usually regarded as the earliest CNN. Since the 21st century, with the proposal of the concept of DL and the continuous improvement of related hardware accelerators and software platforms, CNN has developed rapidly and become one of the most representative algorithms of DL. CNN is most applicable for but is not limited to image processing. To date, CNN has gained widespread applications in many fields, such as computer vision, speech recognition, and NLP.

This paper mainly studies a CNN-based music recommendation system, which further improves the traditional matrix decomposition-based collaborative filtering music recommendation algorithm and fully combines the historical behavior data of users' interaction with music and the acoustic characteristics of music audio. Based on the matrix decomposition of the latent factor model and the CNN regression model with strong feature learning ability, the user and music are projected into a shared hidden space. By calculating the similarity between user preferences and music features, the Top N music recommendation is finally generated for the user. The proposed recommendation algorithm can supplement the information source for the music recommendation system. The overall design block diagram of the system is shown in Figure 2.

As illustrated in Figure 2, the recommendation system includes the following steps:

The first step is to collect the system users' historical behavior data to construct a potential model that can reflect the user-music affinity according to the unified quantitative standard; then, the constructed model is decomposed by the appropriate matrix decomposition method; finally, the implicit vector representation is obtained for user preference features and music features.

The second step is to preprocess the original music resource file and extract the audio feature spectrum of the music.

The third step is to implement a CNN model and take the extracted spectrum as the network input and the music feature vector as the model output (namely, the basic real value of the model). The CNN regression model is finally obtained through continuous training and learning.

The fourth step is to obtain the audio feature spectrum for those newly received music resources; afterward, the CNN regression model can predict the potential features of music, and then based on the user's preference model, the user's music interest is calculated and sorted; finally, Top N new music resources are recommended to relevant users.

Figure 3 demonstrates the proposed CNN network model structure for music potential factor prediction.

Figure 3 shows that the CNN model has four pairs of convolution+pooling layers, in which the convolution layer and pooling layer appear alternately. Finally, there are two full connection layers and one prediction output layer. The input takes the Mel spectrum feature map extracted from the audio, with a pixel size of 256∗256∗1. The convolution operation implements local perception and weight sharing with a convolution step of 2, and the padding = ^“^same^”^ zero is used to fill the matrix edges. The maximum pooling algorithm is adopted with a pooling window of 2∗2. The specific network parameter settings of the convolution layer and full connection layer are shown in Table 1.

In Table 1, *k* represents the potential factor dimension. Here, the effects of different values on the results are compared through experiments. Additionally, to prevent overfitting, the regularization method is to introduce the dropout layer between the full connection layers and set the dropout probability to 50%.

The activation function, loss function, and model error evaluation method are discussed below.

#### 2.4.1. Activation Function

The activation function is usually hidden on the line in the neural network, which can introduce nonlinear factors into the network model so that the model can simulate complex nonlinear functions and deal with more complex logic. If there is no activation function, the neural network is only equivalent to a linear regression model, which cannot represent the complex data distribution. Activation functions feature monotonically differentiable, limited range of output, and nonlinearity and typically include Sigmoid, Tanh, and ReLU. Their equations and function diagrams are shown in Figure 4.

(3) $$\begin{array}{c} \text{Sigmoid}\left(x\right)=\frac{1}{1+{\text{e}}^{-x}}, \end{array}$$

(4) $$\begin{array}{c} \text{ Tanh}\left(x\right)=\frac{e^{x}-e^{-x}}{e^{x}+e^{-x}}, \end{array}$$

(5) ReLUx=max0,x.

Different activation functions will have a distinct impact on the training and prediction of the CNN network model. Compared with Sigmoid and Tanh, ReLU is more widely used in DL; it mainly has the following advantages: first, Sigmoid or Tanh involves a large amount of exponential and division operations and derivation of error gradient by back-propagation, while ReLU activation function can save calculation, which can converge quickly and improve the training efficiency; second, the gradient disappears easily during the back-propagation of Sigmoid function, which makes it impossible to train deep networks, and the gradient of ReLU function is 0 or constant, which can effectively alleviate the problem of gradient disappearance; third, ReLU will make the output of some neurons 0, so it introduces sparsity into the network, and the interdependence between parameters is reduced, which can effectively alleviate overfitting.

Based on the above analysis, this section selects the modified linear unit ReLU as the activation function of the CNN training model.

#### 2.4.2. Loss Function

Supervised learning algorithms generally have an objective function and then optimize it. Usually, the loss function is used as the objective function in the algorithm model dealing with regression or classification tasks. Then, the loss function is used to measure the difference between the predicted value and the real value of the network model output. The main goal of model training is to minimize network loss. The loss function is a nonnegative real value function. The smaller the loss is, the better the performance of the network model is. Meanwhile, different loss functions are usually used to evaluate regression or classification models. Here, the CNN model is used to predict the potential factor characteristics of music audio, which is essentially a regression problem. Therefore, this section only defines the loss function commonly used in the regression model and makes a simple comparison.

Mean Square Error (MSE) loss can be regarded as another calculation method of Euclidean distance, which is defined as follows:

(6) $$\begin{array}{c} \begin{array}{c} \text{Loss}\left(Y,\hat{Y}\right)=\frac{1}{N}\overset{N}{\underset{i=1}{\sum }}{\left({\overset{\wedge }{y}}_{i}-y_{i}\right)}^{2}.\\ \; \end{array} \end{array}$$

Mean Absolute Error (MAE) loss is the average of absolute error of data, which is defined as follows:

(7) $$\begin{array}{c} \begin{array}{c} \text{Loss}\left(Y,\hat{Y}\right)=\frac{1}{N}\overset{N}{\underset{i=1}{\sum }}\left|{\hat{y}}_{i}-y_{i}\right|.\\ \; \end{array} \end{array}$$

Mean Squared Log Error (MSLE) loss is to take the logarithm of the data first and then calculate the Mean Square Error. The definition is as follows:

(8) $$\begin{array}{c} \text{Loss}\left(Y,\hat{Y}\right)=\frac{1}{N}\overset{N}{\underset{i=1}{\sum }}{\left(\log{\overset{\wedge }{y}}_{i}-\log y_{i}\right)}^{2}. \end{array}$$

Mean Absolute Percentage Error (MAPE) loss is defined as follows:

(9) $$\begin{array}{c} \text{Loss}\left(Y,\hat{Y}\right)=\frac{1}{N}\overset{N}{\underset{i=1}{\sum }}\frac{100\times \left|{\hat{y}}_{i}-y_{i}\right|}{y_{i}}. \end{array}$$

Although there are many loss functions to measure the regression model, MSE is still the most widely used loss function; compared with MSE, MAE can effectively punish outliers, which is more suitable for the case of more data outliers; the calculation process of MSLE is similar to that of MSE; its main purpose is to narrow the range of function output values; like MSLE, MAPE is usually used to process a wide range of data, which is to calculate the relative error between the predicted value and the real value. Because this paper will preprocess all the data in advance and normalize the data to a reasonable range and there will not be too many outliers, the MSE is selected as the index to measure the network prediction error. Next, the system experiment and result analysis are carried out.

The dataset acquisition method is as follows. First, 600 songs are randomly downloaded locally through the online music service website and added to the local resource database of the Kugou music client. Then, 12 students are selected as music users. According to the song playing and recording functions of the Kugou music player, the playing time of each song is counted by individual users within 60 days. This way, an available database containing the user's music playing time and the audio file is generated. Afterward, the user's playing data and the audio file are preprocessed accordingly. Importantly, Root Mean Square Error (RMSE) is used to measure the system score's prediction accuracy to verify the experiment. Some datasets are listed in Table 2.

The proposed dataset acquisition method is as follows: firstly, 600 songs are randomly downloaded to the local through the online music service website and added to the local resource database of the Kugou music client. Overall, 12 students are selected as music users based on the song playback and recording function of the Kugou music player, and the playback times are counted for each song by individual users in 60 days. In this way, an available database containing both user music playback times and the audio file is generated, and then the user playback data and audio file are preprocessed accordingly. Root Mean Square Error (RMSE) is used as the measurement standard of prediction accuracy of system score to verify the experiment. The RMSE calculation reads

(10) $$\begin{array}{c} \text{RMSE}=\sqrt{\frac{\sum_{u,ieT}{\left(r_{ui}-{\overset{\wedge }{r}}_{wi}\right)}^{2}}{\left|T\right|}}. \end{array}$$

In Equation ((10)), *T* represents the test dataset, *r*_*ui*_ indicates the real score of user *u* on music *i*, and ${\hat{r}}_{ui}$ stands for the predicted score of the system on music *i*. Equation (11) calculates the accuracy of the recommended list:

(11) $$\begin{array}{c} \text{Precision}=\frac{\sum_{\left.uc\right|}\left|R\left(u\right)\cap T\left(u\right)\right|}{\sum_{ueU}\left|R\left(u\right)\right|}. \end{array}$$

In Equation (11), *R*(*u*) represents the music recommendation list generated by the proposed recommendation system for each user on the test set, and *T*(*u*) denotes all interested music of each user on the test set. The accuracy stands for the proportion that the system-recommended music accepted by users.

The calculation of recall reads

(12) $$\begin{array}{c} \text{Recall}=\frac{\sum_{uel}\left|R\left(u\right)\cap T\left(u\right)\right|}{\sum_{ueU}\left|T\left(u\right)\right|}. \end{array}$$

In Equation (12), the meaning of *R*(*u*) and *T*(*u*) has been defined previously, and the difference between them and the accuracy of calculation lies in the denominator. The recall represents the proportion of proposed system-recommended music in users' actual music selections.

The calculation of the F1 value reads

(13) $$\begin{array}{c} F1=\frac{2PR}{P+R}. \end{array}$$

## 3. Influence of Music Style on the Mental Health of Language-Impaired Students

### 3.1. Case Interview Results

Figure 5 illustrates the qualitative interview results of music imagination, personality, mood, and cognition.

Figure 5 shows that in the qualitative interview results of music imagination, *Fantasia* brings feelings of the sea, childhood, and beautiful melody to language-impaired students, and *Someone Like You* brings about similar experiences, such as love, thanksgiving, and pleasure. In the qualitative interview results of the music personality, the feelings of the language-impaired students brought by *Coming Back Home* are parents, family, and home. In the qualitative interview results of music emotion, *I Believe* brings feelings to the language-impaired students, such as friendship, sandy beach, and breeze, so students can imagine warm pictures with the sound of water and lovers walking hand in hand. In comparison, the feeling brought by *Under the Bodhi Tree* to the language-impaired students is sweet words, such as attachment, affection, and longing. The feelings brought by *Suddenly* to the language-impaired students are crying, breaking up, and helpless, some words about the emotional injury. In the qualitative interview results of music cognition, *Fantasia* brings feelings of quietness, soothing, and nostalgia to language-impaired students, so students can think of their past in this music and find the motivation to move forward. The feelings brought by *Coming Back Home* for the language-impaired students are harmony, coming back home, and missing, so students can yearn for their hometown in this music. The feelings brought by *Electronically synthesized music* to language-impaired students are love, thanksgiving, and beauty, so students can feel the positive energy from this music.

The following are the different music styles: (1) Classical music is a collection of music that possesses the universality of the super-era, eternal artistic value, and the highest performance of music art and acts as the model for the contemporary and future generations. According to this definition, classical music is also called serious music or art music to distinguish it from popular music (pop music). (2) Popular music is a group of commercial music entertainment and related industrial phenomena that focus on marketability rather than artistry. (3) National music, or the so-called Chinese national music, is the assemblage of music created by all ethnic groups from their ancestral life and reproduction in China from ancient times to the present day with cultural tradition, national characteristics, and national spirit. Broadly, Chinese music refers to music with five tones in the world.

### 3.2. The Influence of Music on Negative Emotion

The results of the survey on the music alleviation of *Fantasia*, *Going home*, *I Believe*, and *Under the Bodhi Tree* on negative emotions are shown in Figure 6.

In Figure 6, the independent variable is the negative emotional feelings of the investigated language-impaired students after they are invited to listen to *Fantasia*, *Going home*, *I believe*, and *Under the Bodhi tree*. The dependent variable is the evaluation of alleviation of negative emotions. Multiple regression analysis is conducted, in which *B* is the nonstandardized coefficient. Specifically, the emotional factors that these kinds of music significantly affect (*P* < 0.05) are summarized in Figure 6. The music *Fantasia* can most significantly enhance the three negative emotions of loneliness, anxiety, and fear; the music G*oing home* can most significantly alleviate the four negative emotions: sadness, abomination, loneliness, and anger; the music *I believe* can most significantly enhance pain, loneliness, and complaint, but has the opposite effect on abomination; the music *Under the Bodhi tree* can most significantly enhance sadness, loneliness, and anger, but has the opposite effect on abomination. Additionally, the influence of these kinds of music on other negative emotions is not significant (*P* > 0.05).

Figure 7 presents the QS results of the alleviation effects of *Someone Like You*, *Electronic Synthetic Music*, *Suddenly*, and *Dhyana* from the global music database on negative emotions.

Figure 7 signifies the impact of four different music styles selected from the global music information management database on college students' emotions: *Someone Like You* has the most significant alleviation effect on five negative emotions: anxiety, fear, abomination, sadness, and loneliness; *Electronic Synthetic Music* has the most significant alleviation effect on three negative emotions: loneliness, sadness, and anger, but it stimulates anxiety to a certain extent; *Suddenly* has the most significant alleviation effect on three negative emotions: sadness, loneliness, and complaint; *Dhyana* has the most significant alleviation effect on four negative emotions: pain, loneliness, complaint, and sadness; Additionally, the influence of music emotion recognition model based on Deep Learning (DL) on other negative emotions is not significant (*P* > 0.05) [33].  Figure 8 exhibits the QS analysis results on the alleviation effects of *Vienna Woods Waltz*, *Carmen*, *Remembrance*, and *Balance* from the global music database on negative emotions:

Figure 8 shows the impact of four different music styles selected from the global music information management database on college students' emotions: *Vienna Woods Waltz* has the most significant alleviation effect on three negative emotions: complaint, fear, and sadness; *Carmen* has the most significant alleviation effect on loneliness, sadness, and loneliness; *Remembrance* has the most significant alleviation effect on sadness and pain; *Balance* has the most significant alleviation effect on three negative emotions: pain, loneliness, and anger. Additionally, the influence of music emotion recognition model based on DL on other negative emotions is not significant (**P** > 0.05).  Figure 9 shows the QS analysis results of the alleviation effects of *Waltz of Danube*, *Deep Breathing Freely*, *Harry Potter and the Chamber of Secrets*, and *Blue Love* from the global music database on negative emotions:

Figure 9 demonstrates the impact of four different music styles selected from the global music information management database on college students' emotions: *Waltz of the Danube* has the most significant alleviation effect on two negative emotions: sadness and pain; *Deep Breathing Freely* has the most significant alleviation effect on three negative emotions: sadness, pain, and anger; *Harry Potter and the Chamber of Secrets* has the most significant alleviation effect on four negative emotions: anger, anxiety, fear, and loneliness, but it can stimulate the negative emotion of abomination; *Blue Love* has the most significant alleviation effect on four negative emotions: fear, sadness, loneliness, and anger; additionally, the effect of music emotion recognition model based on DL on other positive emotions is not significant (*P* > 0.05).

### 3.3. The Influence of Music on Positive Emotions

Figure 10 displays the QS results of the enhancement effect of *Fantasia*, *Going home*, *I Believe*, and Under the Bodhi Tree from the global music database on positive emotions:

Figure 10 shows the impact of four different music styles selected from the global music information management database on college students' emotions: *Fantasia* has the most significant enhancement effect on five positive emotions: optimism, incentive, harmony, joy, and hope; *Going home* has the most significant enhancement effect on five positive emotions: optimism, incentive, harmony, joy, hope, and gratitude; *I Believe* has the most significant enhancement effect on five negative emotions: hope, optimism, quietness, incentive, and pride; *Under the Bodhi Tree* has the most significant enhancement effect on five negative emotions: incentive, joy, quietness, hope, and kindness; additionally, the effect of music emotion recognition model based on DL on other positive emotions is not significant (*P* > 0.05).  Figure 11 indicates the QS results of the enhancement effect of *Someone Like You*, *Electronic Synthetic Music*, *Suddenly*, and *Dhyana* from the global music database on college students' positive emotions:

Figure 11 illustrates the impact of different music styles from the global music information management database on college students' emotions: *Someone Like You* has the most significant enhancement effect on six positive emotions: optimism, incentive, harmony, hope, kindness, and pride; *Electronic Synthetic Music* has the most significant enhancement effect on five positive emotions: optimism, pride, hope, harmony, and incentive, but it has a significant inhibition effect on two positive emotions: harmony and joy; the music *Suddenly* has the most significant enhancement effect on six negative emotions: hope, optimism, joy, incentive, and harmony, but it has a significant inhibitory effect on the positive emotion of pride; *Dhyana* has the most significant enhancement effect on five negative emotions: incentive, joy, harmony, quietness, and hope. Additionally, the effect of music emotion recognition model based on DL on other positive emotions is not significant (*P* > 0.05).  Figure 12 displays the findings of the enhancement effect of *Vienna Woods Waltz*, *Carmen*, *Remembrance*, and *Balance* from the global music database on positive emotions:

Figure 12 reveals the impact of four different music styles from the global music information management database on college students' emotions: the music *Vienna Woods Waltz* has the most significant enhancement effect on four positive emotions: optimism, incentive, harmony, and gratitude; *Carmen* has the most significant enhancement effect on six positive emotions: optimism, pride, kindness, quietness, joy, and incentive; *Remembrance* has the most significant enhancement effect on five positive emotions: hope, optimism, joy, incentive, and quietness; *Balance* has the most significant enhancement effect on five positive emotions: incentive, joy, optimism, quietness, and kindness; additionally, the music emotion recognition model based on DL has no significant effect on other positive emotions (*P* > 0.05).  Figure 13 exhibits the QS results on the enhancement effect of *Waltz of the Danube*, *Deep Breathing Freely*, *Harry Potter and Chamber of Secrets*, and *Blue Love* from the global music database on positive emotions:

Figure 13 presents the impact of four different music styles from the global music information management database on college students' emotions: *Waltz of the Danub* has the most significant enhancement effect on six positive emotions: optimism, joy, hope, harmony, gratitude, and pride; *Deep Breathing Freely* has the most significant enhancement effect on seven positive emotions: optimism, quietness, incentive, joy, harmony, gratitude, and kindness; *Harry Potter and Chamber of Secrets* has the most significant enhancement effect on five negative emotions: hope, optimism, hope, incentive, and joy; *Blue Love* has the most significant enhancement effect on of six positive emotions: gratitude, joy, optimism, hope, harmony, and kindness. Additionally, the effect of the music emotion recognition model based on DL on other positive emotions of college students is not significant (*P* > 0.05). Performance analysis of different models on different datasets is shown in Figure 14.

In Figure 14, to further confirm the validity of the proposed effects of music treatment, all the data are statistically analyzed using the factor analysis method. In the single factor model, GFI (Goodness of Fit Index), RMSEA (Root Mean Square Error of Approximation), NNFI (Nonnormed Fit Index), NFI (Normed Fit Index), CFI (Comparative Fit Index), and IFI (Incremental Fit Index) are all lower than the acceptable level, and in the two-factor model, RMSEA > 0.10. The main fitting indexes of the three-factor model CFA of the career planning scale show a high fitting degree and good structural validity. The organizational support scale data factor load is greater than 0.5, and the *t* value is greater than 1.98. The fitting degree of the whole scale model is analyzed. The main fitting indexes of CFA are shown in Figure 14: RMSEA is 0.068, 0.05 ≤ RMSEA ≤ 0.08, indicating that the model fitting is reasonable. The SRMR (Standardized Root Mean Square Residual) = 0.064, less than 0.08, indicating that the whole model is reasonable and has good structural validity.

Robert Schumann has advanced music criticism with his special music review expression. With his rich imagination, keen insight, and true expression of life emotions, Schumann presents various forms of music criticism. He has a strong interest in music and actively uses dialectical thinking to make a judgment on music. His music reviews are sharp and natural, beyond imagination, and he can see things that others generally cannot from different perspectives. Historically, his comments have always resonated with people.

### 3.4. CNN-Based Music Recommendation Algorithm

In this experiment, the Mean Square Error (MSE) is used as the loss function, and the CNN model is trained with the training set data. The training results are shown in Figure 15.

Figure 15 confirms that with the continuous increase of iteration rounds, the loss error of the network model decreases rapidly at the beginning and then gradually becomes slow. When the epoch reaches 10, the error decreases to 0.128, and the function tends to converge. The loss value curve validates that the model's training process basically meets the expected requirements. To better verify the model's prediction ability, the experimental model will be comprehensively evaluated from different angles. The RMSE is used to measure the accuracy of the prediction score. The RMSE results of model prediction scores under different potential factor feature dimensions *k* and training rounds epoch are shown in Figure 16.

Figure 16 certifies that when the *k* is 3 and 5, the RMSE of the prediction score is relatively large, which indicates that the smaller *k* is not enough to represent the potential theme of music; when *k* is 7 and 9, the difference of RMSE of prediction score is not very obvious. The RMSE with *k* = 7 is slightly lower than that with *k* = 9, and in the best case, the RMSE decreases to about 0.6; when *k* = 11, the RMSE of the prediction score begins to increase, which indicates that too large a potential factor dimension will dispel the importance of real potential features. At the same time, with the increase of training rounds, when the epoch is within10-20, the overall RMSE has improved to a certain extent, while the RMSE remains basically unchanged when the epoch is within 20-30, which shows that the preferred training round in this experiment is about 20. After all, a large training round will increase the training time of the whole model. Apparently, when potential factor *k* = 7, and the training round epoch = 20, the experiment can achieve a better score prediction effect, which will lay the basis of the follow-up experiment. Further, experiments are conducted to test the recommendation accuracy under different recommendation list lengths to verify the feasibility of the proposed recommendation algorithm and measure the quality of the recommendation results. In the experiment, the recommended list is set to different lengths, including 10, 15, 20, 25, and 30, respectively, and the accuracy, recall, and F1 value are used to evaluate the accuracy of the recommended list quantitatively. The recommendation results under different recommendation list lengths are shown in Figure 17.

Figure 17 upholds that the length of the recommendation list has a certain impact on the recommendation results, and with the increase of the length of the recommendation list, the accuracy decreases, while the recall and F1 value increase. When the length of the recommendation list is 10, the highest accuracy rate is about 0.41, and the lowest recall is about 0.128. When the length of the recommendation list increases to 30, the accuracy is about 0.31, and the recall rises to about 0.291, which basically conforms to the general law of the recommendation system. The accuracy decreases because the test data are not used for network model training and verification. Hence, the proposed recommendation algorithm has strong prediction and recommendation ability. Then, different algorithms are compared, and the results are shown in Figure 18.

Figure 18 corroborates that under the same recommendation list length, the proposed recommendation algorithm outperforms the other three traditional methods in terms of accuracy, recall, and *F*1 value. This may be because the traditional recommendation algorithms only use a sparse score matrix or a single item content for recommendation, while the proposed recommendation algorithm not only uses the historical behavior data of users' interaction with music but also introduces the features of audio content through DL, and the Deep CNN (DCNN) can better learn the data features.

## 4. Discussion and Suggestions

The structural equation model-fitting implies that music *Fantasy*, *Going home*, *I Believe*, and *Under the Bodhi Tree* have enhanced the positive emotions, which activates the psychosomatic mediation mechanism (nerve excitement, physiological pleasure, and physical and mental relaxation) by 95% and ultimately enhances happiness by 58%, while alleviating pain by 12%. By comparison, *Vienna Woods Waltz*, *Balance*, *Someone Like You*, and *Carmen* have also enhanced positive emotions and alleviated negative emotions, which has activated the psychosomatic mediation mechanism by 83% and eventually enhanced happiness by 67% while alleviating pain by 23%. Thus, music can enhance happiness and alleviate pain by activating psychosomatic mediation mechanisms, which is the significance of the empirical finding here.

The individual's feelings and reactions to the same piece of music vary significantly with personal characteristics. For example, the same song may resonate with someone with its melody or lyrics, while others may show indifference, which is the manifestation of distinct personal feelings. People can be attracted by a musical work for its natural attributes, and most importantly, however, the individual's momentary emotions, physical condition, and life experience, as well as their music preferences, comprehensively affect an individual's music perception (everyone feels out the world through perceptual cognition, and they appreciate music works that can arouse their emotional experience). The empirical study has found that music has a good sublimation effect on people's positive emotions. Specifically, different music personality traits can enhance various dimensions of positive emotions; different music styles can enhance the positive emotions independently; different music styles can enhance the same positive emotions.

Classical music manifests more than a classical atmosphere but has unique high attainments in music connotation. Meanwhile, classical music is often featured by regional religions and humanities and creates an elegant, noble, mysterious, and holy ambiance. Moreover, classical music enhances love and gratitude and encourages upward personality quality. Such music stimulates people's positive emotions for the pursuit of truth, goodness, and beauty so that the soul gets deeper sublimation. In short, classical romantic music can stimulate people's *s* positive emotions. Popular music is the simplest musical form with the most extensive propagation and catching lyrics. Popularity is the art of speaking. When appreciating popular music, people are more deeply aware of the reality and intimacy of the music. In music style, composition form, and presentation form, popular music is completely different from classical music. For the emerging forms of artistic expression, impromptu accompaniment singing music can better adjust the atmosphere of the scene, touch the listeners' hearts, enrich their imagination, and promote their psychosomatic health. The original ecological music of ethnic minorities exerts a unique exotic flavor, inheriting the essence of traditional culture, developing its unique style, and radiating special artistic charm. Hence, various styles of music play different roles in music intervention experiments, in which listeners experience astral joviality and musical imagination. To sum up, the positive effect of music can improve people's positive psychology.

## 5. Conclusion

Under the social background of increasingly fierce competition, language-impaired students' psychological pressure increases and becomes an important social issue. This work analyzes language-impaired students' psychological reactions to different music styles, such as emotional response and audiovisual synaesthesia. It also studies students' recognition and selection of music styles to explore ways to alleviate their psychological pressure. The main conclusions are as follows. (1) Different music creation styles generate significantly different emotional responses to the same subject, and the music performance is consistent with the actual feelings of the subjects. (2) Different music styles cause different associations in students' minds, leading to different psychological reactions. Soft and relaxing music has the most significant effect on relieving students' learning pressure, compared to music with a strong sense of rhythm and vitality, which has little effect. (3) The music recommendation model based on CNN can assist music psychotherapy well. Last but not least, although the research subject has been fully considered, there are still some deficiencies. Most notably, the music style studied has great limitations. Therefore, in future research, the music database should be further expanded with the development of information globalization technology, and a more comprehensive music style should be used to study the mental health status of language-impaired college students.

## Figures and Tables

**Figure 1:** Structure equation prediction model diagram.

**Figure 2:** Overall design block diagram of music recommendation system based on CNN.

**Figure 3:** CNN model structure for music potential factor prediction.

**Figure 4:** Schematic diagram of several common activation functions.

**Figure 5:** The results of qualitative interviews of music ((a) imagination; (b) personality; (c) mood; (d) cognition).

**Figure 6:** The survey results of the music alleviation on negative emotions (the vertical coordinate *B* represents the nonstandardized coefficient, which shares the same as that in the following figures. (a) *Fantasia*; (b) *Going home*; (c) *I believe*; (d) *Under the Bodhi tree*).

**Figure 7:** QS results of alleviation effects of different music styles on negative emotions around the world ((a) regression analysis of *“someone like you”*; (b) regression analysis of *“Electronic Synthetic Music”*; (c) regression analysis of *“Suddenly”*; (d) regression analysis of *“Dhyana”*; *B* represents the nonstandardized coefficient; *t* denotes the emotional factor).

**Figure 8:** QS results of alleviation effects of different music styles on negative emotions around the world ((a) *“Vienna Woods Waltz”*; (b) *“Carmen”*; (c) *“Remembrance”*; (d) *“Balance”*; *B* represents nonstandardized coefficient; *t* is the emotional factor).

**Figure 9:** QS results on the alleviation effects of different music styles on negative emotions around the world ((a) *“Waltz of the Danube”*; (b) *“Deep Breathing Freely”*; (c) *“Harry Potter and the Chamber of Secrets”*; (d) *“Blue Love”*; *B* is the nonstandardized coefficient; *t* represents the emotional factor).

**Figure 10:** QS results of the enhancement effect of different music styles on positive emotions around the world ((a) *“Fantasia”*; (b) *“*G*oing home”*; (c) *“I believe”*; (d) *“Under the Bodhi Tree”*; *B* is the nonstandardized coefficient; *t* represents the emotional factor).

**Figure 11:** QS results in the enhancement effects of different music styles on positive emotions around the world ((a) *“Someone Like You”*; (b) *“Electronic Synthetic Music”*; (c) *“Suddenly”*; (d) *“Dhyana”*; *B* is the nonstandardized coefficient; *t* represents the emotional factor).

**Figure 12:** QS results of enhancement effects of different music styles on positive emotions around the world ((a) *“Vienna Woods Waltz”*; (b) *“Carmen”*; (c) *“Remembrance”*; (d) *“Balance”*; *B* is nonstandardized coefficient; *t* stands for the emotional factor).

**Figure 13:** QS results of enhancement effects of different music styles on positive emotions around the world ((a) *“Waltz of the Danube”*; (b) *“Deep Breathing Freely”*; (c) *“Harry Potter and Chamber of Secrets”*; (d) *“Blue Love”*; *B* is the nonstandardized coefficient; *t* denotes emotional factor).

**Figure 14:** Model fitting test results ((a) comparison of the main fitting indexes of the type I music CFA (Color Filter Array); (b) comparison of the main fitting indexes of type II music CFA; (c) comparison of the main fitting indexes of the type III music CFA; (d) comparison of the main fitting index of type IV music CFA).

**Figure 15:** Training model loss curve.

**Figure 16:** Model training prediction score for RMSE.

**Figure 17:** Recommendation results under different recommendation list lengths.

**Figure 18:** Comparison of different recommendation algorithm models ((a) accuracy; (b) recall; (c) *F*1 value).

**Table 1:** Parameters of the CNN model.

Convolutional layer	Convolution kernel size	Number of convolution kernels
1	3 × 3	64
2	3 × 3	128
3	2 × 3	256
4	2 × 3	512
Full connection layer	Number of input	Number of outputs
1	512	128
2	128	32
3	32	k

**Table 2:** Partial dataset trained in CNN model.

Training set		Test set	
Music name	Music playing time	Music name	Music playing time
The lone brave	2365411.31 h	Strange fire	4126358.26 h
Blossom all the way	1255485.37 h	Madame Butterfly	215687.126 h
Days after the next stop	1426358.75 h	Spare no time	1569774.89 h
Three lives and three blessings	954631.21 h	WHO	179643.45 h
Mom's words	914568.32 h	Invisible Man	1423586.16 h

## Data Availability

All data are fully available without restriction.
